The article "Prenatal Cocaine Exposure Uncouples mGluR1 from Homer1 and Gq Proteins" was retracted in 2022. Reasons: concerns about the data; concerns about the images.

# Prenatal Cocaine Exposure Uncouples mGluR1 from Homer1 and Gq Proteins

**DOI:** 10.1371/journal.pone.0091671

**Published:** 2014-03-13

**Authors:** Kalindi Bakshi, Raminder Parihar, Satindra K. Goswami, Melissa Walsh, Eitan Friedman, Hoau-Yan Wang

**Affiliations:** Departments of Physiology, Pharmacology and Neuroscience, Sophie Davis School of Biomedical Education, The City University of New York Medical School, New York, New York, United States of America; University of Colorado, United States of America

## Abstract

Cocaine exposure during gestation causes protracted neurobehavioral changes consistent with a compromised glutamatergic system. Although cocaine profoundly disrupts glutamatergic neurotransmission and *in utero* cocaine exposure negatively affects metabotropic glutamate receptor-type 1 (mGluR1) activity, the effect of prenatal cocaine exposure on mGluR1 signaling and the underlying mechanism responsible for the prenatal cocaine effect remain elusive. Using brains of the 21-day-old (P21) prenatal cocaine-exposed rats, we show that prenatal cocaine exposure uncouples mGluR1s from their associated synaptic anchoring protein, Homer1 and signal transducer, Gq/11 proteins leading to markedly reduced mGluR1-mediated phosphoinositide hydrolysis in frontal cortex (FCX) and hippocampus. This prenatal cocaine-induced effect is the result of a sustained protein kinase C (PKC)-mediated phosphorylation of mGluR1 on the serine residues. In support, phosphatase treatment of prenatal cocaine-exposed tissues restores whereas PKC-mediated phosphorylation of saline-treated synaptic membrane attenuates mGluR1 coupling to both Gq/11 and Homer1. Expression of mGluR1, Homer1 or Gα proteins was not altered by prenatal cocaine exposure. Collectively, these data indicate that prenatal cocaine exposure triggers PKC-mediated hyper-phosphorylation of the mGluR1 leading to uncoupling of mGluR1 from its signaling components. Hence, blockade of excessive PKC activation may alleviate abnormalities in mGluR1 signaling and restores mGluR1-regulated brain functions in prenatal cocaine-exposed brains.

## Introduction

Cocaine usage during pregnancy causes protracted neurological and behavioral abnormalities [1]–[3]. Although prenatal cocaine exposure alters glutamatergic function in various brain regions [4]–[6], the effect of gestational cocaine exposure on metabotropic glutamate receptor (mGluR) is not well understood. Recently, prenatal cocaine exposure was shown to directly disrupt mGluR1 function resulting in delays in postnatal synaptic maturation [7].

The mGluRs are members of the G-protein coupled receptor (GPCR) superfamily that modulate neuronal excitability and development, synaptic plasticity and neurotransmitter release underlying optimal cognitive function [8]. There are eight members in the mGluR family that are divided into three groups: group I – mGluR1 and 5, group II – mGluR2 and 3, group III – mGluR [4,] [6]–[9]. The group I mGluRs (mGluR1 and mGluR5) are coupled exclusively to Gq/11 to regulate phospholipase C and inositol 1,4,5-tris phosphate (IP_3_) receptors through their association with a constitutively expressed synaptic scaffolding protein, Homer1 [10]–[12]. Group 1 mGluRs are predominantly expressed in the postsynaptic somatodendritic regions, especially in brain areas highly responsive to psychostimulants including Nucleus accumbens (NAc), whereas Groups II and III mGluRs are mainly localized presynaptically on axons and axonal terminals [13], [14].

Prenatal cocaine exposure produces long-lasting cognitive deficits in humans and animal models [15], [16]. Since mGluR1 is a pivotal regulator of the glutamatergic neurotransmission and cognitive processes, it is highly conceivable that prenatal cocaine exposure induces cognitive defects through alterations in the mGluR1 signaling. This hypothesis may be supported by the data showing that repeated cocaine exposure produces a persistent reduction in mGluR function in the NAc after a three week withdrawal period [17]. This cocaine-mediated effect was attributed to a decrease in, or complete deletion of Homer1, a pivotal synaptic anchoring protein for group 1 mGluRs that modulates IP_3_ production and intracellular Ca^2+^ mobilization [12], [17], [18]. In line with the notion that prenatal cocaine exposure affects mGluR1 function, delay in synaptic maturation in prenatal cocaine exposed brains was attributed in part to the impaired mGluR1 function [7]. Together, these data lead us to thoroughly study the effect of *in utero* cocaine exposure on mGluR1-mediated signaling in frontal cortex (FCX) and hippocampus, two brain regions vital for cognitive function, in the rat prenatal cocaine model. We further identify the underlying mechanism through which prenatal cocaine exposure elicits signaling dysfunction in the mGluR1 system.

## Materials and Methods

### Materials and Chemicals

Soybean trypsin inhibitor, phenylmethylsulfonyl fluoride [PMSF], 2-mercaptoethanol, NaF, Na_2_VO_4_, Digitonin, protein phosphatase inhibitor I & II cocktails, recombinant γPKC, alkaline phosphatase, phorbol 12-myristate, 13-acetate (PMA), anti-phosphoserine (P3430), anti-phosphothreonine (P3555) were purchased from Sigma (St. Louis, MO). Leupeptin and aprotinin were from Peptide International (Louisville, KY). Phorbol 12-myristate, 13-acetate (PMA) was from Enzo Life Science (Plymouth Meeting, PA). Antibody against mGluR1 was purchased from Transduction Laboratories (Madison, WI). (S)-3,5-dihydroxyphenylglycine (DHPG), α-Amino-5-carboxy-3-methyl-2-thiopeneacetic acid (3-MATIDA) were purchased from Tocris Bioscience (Minneapolis, MN). Antibodies against phosphotyrosine (SC-508), caspase-3 (SC-7272), β-actin (SC-47778), Homer1 (SC-55463), Homer2 (SC-8924), Gαs/olf (SC-383), Gαi (SC-7276), Gαo (SC-387) or Gαq/11 (SC-392), actin (SC-1616R) were purchased from Santa Cruz Biotechnology (Santa Cruz, CA). Immobilized protein A/G-conjugated agarose, Seize-X immunoprecipitation kit, antigen elution buffer and West pico chemiluminescent reagents were purchased from Thermo Pierce (Rockford, IL). Celestrine was purchased from EMD Cal-Biochem (La Jolla, CA). Bradford reagent, SDS-PAGE reagents, pre-stained molecular weight markers were purchased from Bio-Rad (Hercules, CA). 10-KDa cut-off filters were obtained from Cole-Palmer (Vernon Hills, IL).

### Animals

Pathogen-free, 10-week-old male and female Sprague-Dawley rats weighing approximately 200–215 g (Taconic, Germantown, NY) were housed individually in a 12-hr light/dark cycle with free access to food and water. All animal procedures were in compliance with the National Institutes of Health *Guide for Care Use of Laboratory Animals* and were approved by the City College of New York Animal Care and Use Committee. The animal treatment was performed as described previously [6]. Briefly, pregnant dams were assigned to receive daily intraperitoneal (ip) injections from GD 8–20 of either cocaine HCl, 30 mg/kg in 0.9% saline or saline, 2 ml/kg. The animals were injected daily between 9–10 AM. Following each injection, these pregnant rats were observed for 1 hr and behavioral abnormalities recorded. There were no discernible differences in litter size (between 7–13 pups) and body weight of the pups at 21-day of age (47.5±3.1 and 52.7±2.4 g for cocaine and saline, respectively; *n* = 30 each) and gender distribution (17 males/13 females and 14 males/16 females for cocaine and saline groups, respectively). There were no obvious changes in rearing behaviors. Importantly, the dose of cocaine used did not induce seizure or fatality throughout the treatments.

The progenies were cross-fostered to a naïve mother until sacrificed at 21 days of age (P21). They were subjected to the minimum handling associated with routine animal husbandry. Importantly, we did not find gender differences in our previous studies conducted in rabbit and rats [5], [6], [19], [20], both sexes from separate litters were employed in these experiments. To avoid the pitfall from oversampling [21], only one animal from each litter was used in each experiment reported here. Pups were sacrificed by rapid decapitation, the brains removed immediately on ice, and coronal cuts at optic chiasm and +4 mm rostral to optic chiasm were made to dissect out the FCX and prefrontal cortex. To minimize skin lesions in the cocaine-injected rats, the injection sites were alternated every other day.

### Preparation of Synaptosome and Fractionation

Synaptosomes (P2 fraction) were prepared from frontal cortices as previously described previously with few modifications [22], [23]. To further purify synaptosomal factions, the synaptosome-enrich P2 fraction was washed twice in 5 ml of oxygenated ice-cold Kreb’s-Ringer solution (K-R): 25 mM HEPES, pH 7.4; 118 mM NaCl, 4.8 mM KCl, 25 mM NaHCO_3_, 1.3 mM CaCl_2_, 1.2 mM MgSO_4_, 1.2 mM KH_2_PO_4_, 10 mM glucose, 100 µM ascorbic acid, 50 µg/ml leupeptin, 10 µg/ml aprotinin, 2 µg/ml soybean trypsin inhibitor, 0.04 mM phenylmethylsulfonyl fluoride (PMSF), 0.1 mM 2-mercaptoethanol, 10 mM NaF, 1 mM Na_3_VO_4_ and 0.5 µl/ml protein phosphatase inhibitor I & II cocktails (Sigma, St. Louis, MO). To obtain cytosolic and membranous fractions of the synaptosomes, the washed synaptosomes were sonicated for 10 sec on ice in 0.5 ml hypo-tonic homogenization solution (25 mM HEPES, pH 7.4; 12 mM NaCl, 0.5 mM KCl, 2.5 mM NaHCO_3_, 0.1 mM CaCl_2_, 0.1 mM MgSO_4_, 0.1 mM KH_2_PO_4_, 1 mM glucose, 10 µM ascorbic acid, 50 µg/ml leupeptin, 10 µg/ml aprotinin, 2 µg/ml soybean trypsin inhibitor, 0.04 mM PMSF and 0.1 mM 2-mercaptoethanol, 10 mM NaF, 1 mM Na_2_VO_4_ and 0.5 µl/ml protein phosphatase inhibitor I & II cocktails). Samples were then centrifuged at 50,000×g for 30 min. The resultant supernatant was taken as cytosolic fraction and synaptic membrane pellet was resuspended in 0.5 ml of K-R solution. Protein concentrations of the synaptic membranes were determined using the Bradford method (Bio-Rad) and used as the tissue source for determination of the levels of mGluR1-G protein-Homer1 coupling.

### *In vitro* Determination of mGluR1 - G Protein and -Homer1 Interaction and Immunoprecipitation

To assess the effect of prenatal cocaine exposure on mGluR1 - G protein and -Homer1 coupling, synaptic membranes (200 µg) derived from frontal cortices and hippocampi of 21-day-old rats that were exposed to either saline or cocaine during gestation were incubated with 1 µM glutamate or K-R for 5 min at 37°C (total incubation volume: 250 µl). Following incubation, 750 µl Ca^2+^-free K-R containing 0.5 mM EGTA was added and synaptic membranes were pelleted by centrifugation. Synaptic membranes were then solubilized by brief sonication (10 sec, 50% output, Fisher Scientific) in 250 µl of immunoprecipitation buffer (25 mM HEPES, pH 7.5; 200 mM NaCl, 1 mM EDTA, 50 µg/ml leupeptin, 10 µg/ml aprotinin, 2 µg/ml soybean trypsin inhibitor, 0.04 mM PMSF, 5 mM NaF, 1 mM sodium vanadate, 0.5 mM β-glycerophosphate and 0.1% 2-mercaptoethanol containing 0.5% digitonin, 0.2% sodium cholate and 0.5% NP-40 and incubated at 4°C with end-to-end shaking for 1 hr. Following dilution with 750 µl of ice-cold immunoprecipitation buffer and centrifugation at 4°C to remove insoluble debris, the resultant lysate was used to identify and measure the effect of prenatal cocaine exposure on mGluR1-G_q/11_-Homer1 interaction.

To identify the G protein(s) associated with mGluR1, we used co-immunoprecipitation of mGluR1 with specific G protein(s). Briefly, frontal cortical and hippocampal lysates from control rats were immunoprecipitated with 1 µg immobilized anti-Gαs/olf, - Gαi, - Gαo or - Gαq/11 for 16 hr incubation at 4°C as described previously [24]. Following centrifugation, the obtained anti-Gα immunoprecipitates were washed three times with 1 ml of ice-cold phosphate-buffered saline, pH 7.2 (PBS), the isolated mGluR1/G protein signaling complexes were solubilized by boiling for 5 min in 100 µl of SDS-PAGE sample preparation buffer (62.5 mM Tris-HCl, pH 6.8; 10% glycerol, 2% SDS; 5% 2-mercaptoethanol, 0.1% bromophenol blue). The presence of mGluR1 was detected by Western blotting with anti-mGluR1 together with anti-Gαafter size-fractionation of the solubilized anti-Gα immunoprecipitate to confirm the presence of mGluR1 and indicated Gα proteins.

In addition, synaptic membranes were incubated with 1 µ M glutamate at 37°C for 5 min. The reaction was terminated by addition of ice-cold 20 mM Mg^2+^-containing K-R. The synaptic membranes were then collected by centrifugation and solubilized as described above. The obtained membranous lysate was immunoprecipitated with 1 µg of either immobilized anti-mGluR1 followed by 30 µl immobilized protein A/G-conjugated agarose. The resultant anti-mGluR1 immunoprecipitates was probed with anti-Gαq and Homer1 using Western blotting.

To determine the effect of prenatal cocaine exposure on the mGluR1-G_q/11_-Homer1 linkages, mGluR1-G_q/11_-Homer1 complexes in frontal cortical and hippocampal synaptic membrane lysates from prenatal saline- and cocaine-exposed rats were isolated by immunoprecipitation for 16 hr incubation at 4°C with 1 µg of immobilized anti-mGluR1- protein A-conjugated agarose beads. The resultant immunocomplexes were pelleted by centrifugation at 4°C. After three washes with 1 ml of ice-cold PBS and centrifugation, the isolated mGluR1 signaling complexes were solubilized by boiling for 5 min in 100 µl of SDS-PAGE sample preparation buffer. Following brief centrifugation to remove immobilized antibody-protein A/G agarose complexes, the levels of G_q/11_-mGluR1 and mGluR1-Homer1 association were estimated by the amount of Gα_q/11_ and Homer1 in anti-mGluR1 immunoprecipitates by Western blotting. Equal loading of the anti-mGluR1 immunoprecipitates was confirmed by Western blotting that assessed the amount of mGluR1.

In the experiments where the phosphorylation state of mGluR1 was assessed, frontal cortical synaptic membranes (100 µg) from prenatal saline- and cocaine-exposed rats were suspended in K-R without protein phosphatase inhibitors. Membranes were incubated with 100 µg/ml alkaline phosphatase in Tris, pH 8.0, 130 mM NaCl, protease inhibitors at 30°C for 20 min (total incubation volume 100 µl). The phosphatase activity was terminated by adding 10 mM NaF/1 mM Na_3_VO_4_. To assess the effect of specific PKC-mediated phosphorylation, dephosphoryated membranes from saline-treated P21 rats was incubated with 0.5 µg/ml recombinant γPKC, 20 µg phosphotidylserine and 162 nM phorbol 12-myristate, 13-acetate (PMA) in the presence of 30 µM ATP in K-R at 30°C for 10 min (total incubation volume 125 µl). The actions of PKC were terminated by addition of 1 µM celestrine. Following termination of the reaction, membranes were incubated with K-R or 1 µM glutamate at 37°C for 5 min. The reaction was stopped by adding 375 µl of ice-cold Ca^2+^-free K-R containing 0.5 µM EGTA and synaptic membranes were collected by centrifugation. The obtained synaptic membrane pellet was immediately solubilized by brief sonication in immunoprecipitation buffer with 0.5% digitonin, 0.2% sodium cholate and 0.5% NP-40 and incubated at 4°C with end-to-end shaking for 1 hr. Following dilution with 750 µl of ice-cold immunoprecipitation buffer and centrifugation at 4°C to remove insoluble debris, the mGluR1-G_q/11_-Homer1 complexes were co-immunoprecipitated using 1 µg immobilized anti-mGluR1 protein A-agarose beads overnight at 4°C. The immunoprecipitate was pelleted by centrifugation and washed 3 times each with 1 ml PBS. The mGluR1-G_q/11_-Homer1 complexes were eluted with 75 µl of antigen elution buffer (Pierce). The eluate containing mGluR1-G protein-Homer1 was immediately neutralized by 10 µl 1.5 M Tris, pH 8.8 and 15 µl 6X sample preparation buffer was added. After boiling for 5 min, phosphor-serine, -threonine and -tyrosine content in mGluR1 was sequentially analyzed by Western blotting with antibodies directed against phosphoserine first (anti-phosphoserine), stripped and re-probed three times sequentially with anti-phosphothreonine, -phosphotyrosine and then -mGluR1. The signals were detected using a chemiluminescent method and visualized by exposure to x-ray film for 5–30 sec. Specific protein bands were quantified by densitometric scanning (GS-800 calibrated densitometer, Bio-Rad Laboratories).

### Western Blotting

To determine whether prenatal cocaine exposure influences the expression of mGluR1, Homer1 or various Gα proteins, synaptic membranes of frontal cortices and hippocampi from 21-day-old prenatal saline- and cocaine-exposed rats were boiled for 5 minutes in 100 µl PAGE sample buffer and then size fractionated on 10% SDS-PAGE. Proteins were transferred to nitrocellulose membrane and Western blotting was performed with antibodies for mGluR1, Homer-1, phosphotyrosine, phosphoserine, phosphothreonine, Gαs/olf, Gαi, Gαo or Gαq/11. The blots were stripped and re-probed with anti-actin, anti- Gα (co-immunoprecipitation of mGluR1– G protein), anti-mGluR1 (co-immunoprecipitation of mGluR1 - Homer1 and -G_q/11_ or phosphorylated mGluR1) to verify equal sample loading and immunoprecipitation efficiency.

Immunoreactivity was detected by a chemiluminescent method and visualized by immediately exposing to X-ray film for 10–30 sec. Specific protein bands were quantified by densitometric scanning (GS-800 calibrated densitometer, Bio-Rad Laboratories).

### Measurement of IP_3_ Accumulation

The effect of prenatal cocaine on mGluR1-mediated IP_3_ accumulation was determined in frontal cortical and hippocampal slices from P21 prenatal cocaine- and saline-exposed rat brains using an established method with slight modifications [25]. Brain tissues were brought to room temperature in oxygenated K-R, pH 7.4. The tissues were chopped into 350×350 µm slices, washed twice with K-R at room temperature and incubated for 15 min in K-R followed by 30 min with 1 µM (S)-3,5-dihydroxyphenylglycine (DHPG) or K-R at 37°C in a shaking water bath. The slices were then washed twice with pH 7.0 hypotonic buffer containing 20 mm Tris-HCl, 1 mM EGTA at 4°C. The slices were collected by brief centrifugation and homogenized in 1.5 ml of 1 M trichloroacetic acid (TCA) using 10 hand strokes of a Teflon-glass homogenizer. Homogenates were then placed on ice for 15 min before centrifugation at 13,000 *g* for 10 min. The resultant pellets were washed three times with distilled H_2_O and digested in 1 M NaOH and the protein levels were determined using Bradford method (Bio-Rad). The specificity of DHPG was assessed by pretreatment of the slices with 10 µM α-Amino-5-carboxy-3-methyl-2-thiopeneacetic acid (3-MATIDA). One ml of trichloro trifluoro ethan-trioctylamine (3∶1) was added to 500 µl of TCA tissue extract in a polypropylene eppendorf tube, mixed vigorously for 15 sec and then centrifuged for 1 min at 10,000 g. Aliquots of the upper phase were taken for IP_3_determination according to the instructions from the manufacturer of the assay kit (PerkinElmer). The IP_3_ concentrations are expressed as pmol/mg protein.

### Data Analysis and Statistical Evaluation

Statistical differences between cocaine and saline groups were assessed using the two-tailed Student’s *t* test.

## Results

### Prenatal Cocaine Exposure Uncouples mGluR1 from Gq/11 and Homer1

We first assess whether mGluR1s are coupled to specific G protein(s). The data shown in Fig. 1A illustrates that mGluR1 is coupled exclusively to Gq/11 and exposure to 1 µM glutamate increases mGluR1 - Gq/11 coupling by approximately 4.5-fold in both FCX and hippocampus. In addition, mGluR1 - Gq/11 complex is associated with scaffolding protein Homer1 but not Homer2 (data not shown) as both Gαq/11 and Homer1 were detected in anti-mGluR1 immunoprecipitate in both brain regions (Fig. 1B). Unlike the coupling of mGluR1 to Gq/11, glutamate stimulation did not affect mGluR1-Homer1 association. The effect of prenatal cocaine exposure on the association of mGluR1 with Gq/11 and Homer1 was subsequently determined by the level of Gαq/11 and Homer1 co-immunoprecipitated with mGluR1. The data summarized in Fig. 2 show that prenatal cocaine exposure markedly reduces the levels of mGluR1 coupling to Homer1 by 56.0±4.9–57.8±10.1% and glutamate-induced but not basal mGluR1 coupling to Gq/11 by 69.0±12.3 - 63.4±3.2% in both FCX and hippocampus. This prenatal cocaine effect was not caused by alteration in the mGluR1, Gα or Homer1 expression as comparable levels of these proteins were noted in both brain regions examined (Fig. 3).

**Figure 1:** The mGluR1 is associated exclusively with G_q/11_ and Homer1 in the frontal cortex (FCX) and hippocampus of 10-week-old naïve rats. (**A**) The presence of mGluR1 was examined in the immobilized anti-Gα immunoprecipitates of the solubilized FCX and hippocampal synaptosomal membranes by Western blotting. The representative Western blots show exclusive detection of mGluR1 together with Gαq/11 protein in the synaptosomes prepared from FCX and hippocampus. N = 4. (**B**) Basal and glutamate (1 µM)-induced mGluR1 coupling to G_q/11_ and Homer1 in synaptic membranes derived from FCX and hippocampi of 10-week-old naïve rats. The presence of mGluR1 was examined in immobilized anti-mGluR1 immunoprecipitates of the solubilized FCX and hippocampal synaptosomal membranes by Western blotting. The representative Western blots show Gαq/11 protein and Homer1 are present in anti-mGluR1 immunoprecipitates. Quantitative data are presented as means ± s.e.m. of the ratios of optical intensity of indicated protein to the optical intensity of mGluR1 (2132.8±150.8 and 2090.8±151.8 optical intensity in FCX of Kreb’s-Ringer (K-R) and glutamate treated, respectively and 2044.5±139.2 and 2000.0±114.3 optical intensity in hippocampi of K-R and glutamate treated, respectively) to validate equal loading. There is no discernible difference in the level of mGluR1-associated Homer1 indicated as Homer1/mGluR1 ratios in both brain regions (0.467±0.03 vs. 0.447±0.03 in K-R and glutamate exposed FCX and 0.468±0.03 vs. 0.488±0.02 in K-R and glutamate exposed hippocampus). Incubation with 1 µM glutamate increased the level of Gq/11 associated with mGluR1 by 343.2±28.9% and 332.7±32.1% respectively in FCX and hippocampus. *N* = 4 for each group. *p<0.01 comparing the level of Gαq/11 in K-R and 1 µM glutamate exposed synaptosomal membranes by two-tailed Student’s *t* test.

**Figure 2:** Prenatal cocaine exposure markedly reduces mGluR1 association with G_q/11_ and Homer1 in the FCX and hippocampus of P21 rats. (**A**) The levels of G_q/11_ and Homer1 associated with mGluR1s were examined in the immobilized anti-mGluR1 immunoprecipitates of the solubilized FCX and hippocampal synaptosomal membranes of prenatal saline- and cocaine-exposed P21 rats following incubation with Kreb’s-Ringer (K-R) or 1 µM glutamate by Western blotting. The representative Western blots show the detection of Gα_q/11_ protein and Homer1 in the synaptosomal membranes prepared from FCX and hippocampus. Glutamate increased mGluR1 coupling to G_q/11_ but not to Homer1. N = 4. (**B**) Quantitative data are presented as means ± s.e.m. of the ratios of optical intensity of indicated protein to the optical intensity of mGluR1 (1894.3±122.1–2068.8±348.3 optical intensity in FCX of saline and cocaine, respectively and 185.1±99.9–1885.5±98.3 optical intensity in hippocampi of saline and cocaine, respectively) to validate equal loading. Incubation with glutamate increased G_q/11_ - mGluR1 coupling by 298.8±33.9% and 387.2±31.4% in FCX and hippocampus respectively. This glutamate-induced G_q/11_-mGluR1 coupling was reduced by 69.0±12.3% and 63.4±3.2% respectively in FCX and hippocampus. Glutamate did not alter Homer1-mGluR1 coupling, whereas prenatal cocaine exposure reduced Homer1-mGluR1 association by 56.0±4.9–57.8±10.1% and 52.6±8.0–55.1±10.4% respectively in FCX and hippocampus. N = 4 for each group. *p<0.01, **p<0.05 comparing the level of Gαq/11 in K-R and 1 µM glutamate exposed brain synaptosomal membranes by two-tailed Student’s *t* test. #*p*<0.01 comparing the G_q/11_ - mGluR1 or Homer1 - mGluR1 coupling levels in cocaine- to saline-treated groups by two-tailed Student’s *t* test.

**Figure 3:** Prenatal cocaine exposure did not alter the expression of various Gα proteins, Homer1 and mGluR1 in the FCX and hippocampus of P21 rats. (**A**) Representative Western blots of the Gα proteins, Homer1 and mGluR1 in the FCX and hippocampal synaptosomes of P21 rats exposed to saline or cocaine during gestation. The blots were stripped and sequentially re-probed with anti-actin (2265.5±129.9 and 2378.8±174.8 optical intensity in FCX of saline and cocaine, respectively and 2160.5±104.8 and 2125.0±131.7 optical intensity in hippocampi of saline and cocaine, respectively) to validate equal loading. (**B**) Densitometric quantification of the Gα proteins, Homer1 and mGluR1 levels in the FCX and hippocampus of P21 rats. Data are presented as means ± s.e.m. of the ratios of optical intensity of indicated protein to the optical intensity of actin. *N* = 4 for each group. There are no discernible changes in the expression levels of any of the proteins examined in either brain regions of the prenatal cocaine exposed rats.

### Prenatal Cocaine Exposure Attenuates mGluR1-mediated IP_3_ Accumulation

To assess the impact of prenatal cocaine exposure on mGluR1-mediated function, we measured the level of IP_3_ induced by 1 µM DHPG, a group I mGluR specific agonist. Our results summarized in Fig. 4 indicate that prenatal cocaine reduces DHPG-induced IP_3_ accumulation in the FCX and hippocampus. Pretreatment with mGluR1-specific antagonist, 3-MATIDA resulted in an approximately 65–70% in both brain regions (data not shown). In both brain areas from P21 prenatal cocaine-exposed rats, a 52.0±6.9–62.6±8.4% reduction in DHPG-elicited IP_3_ accumulation without alteration in basal IP_3_ level were noted (Fig. 4).

**Figure 4:** Prenatal cocaine exposure markedly reduces mGluR1-induced phosphoinositide hydrolysis in the FCX and hippocampus of P21 rats. The levels of 1 µM DHPG induced IP_3_ accumulation was measured using an assay kit according to manufacturer’s instructions. Prenatal cocaine exposure did not affect the basal IP_3_ levels in FCX (12.03±0.93 vs. 11.71±0.93 pmol/mg protein in saline and cocaine, respectively) and in hippocampus (11.95±1.26 vs. 12.71±1.63 pmol/mg protein in saline and cocaine, respectively). Incubation with 1 µM DHPG resulted in a 137.0±8.7% and a 41.2±10.2% increase in IP_3_ levels in FCX and hippocampus, respectively. Prenatal cocaine exposure markedly reduced DHPG-induced phosphoinositide hydrolysis by 52.0±6.9–62.6±8.4% in both brain regions. Data are presented as means ± s.e.m. of the IP_3_ level in pmol/mg protein. *N* = 6 for each group. *p<0.01, **p<0.05 comparing the IP_3_ level in Kreb’s-Ringer and 1 µM DHPG exposed brain tissues by two-tailed Student’s *t* test. #*p*<0.01 comparing DHPG-induced IP_3_ in cocaine to saline-treated group by two-tailed Student’s *t* test.

### Prenatal Cocaine Exposure Increases Serine-phosphorylation of the mGluR1

To identify the mechanism responsible for uncoupling of the mGluR1 from its associated G_q/11_ protein and Homer1, we considered alteration in the phosphorylation state of the mGluR1 since altered phosphorylation state of the receptor can result in receptor - G protein dissociation [26]. The data shown in Fig. 5A indicate that the level of phosphoserine (pS) in mGluR1 was increased by 150.8±9.2% and 143.4±9.5% exclusively in FCX and hippocampus of prenatal cocaine-exposed brains, respectively.

**Figure 5:** Serine phosphorylation of mGluR1 is elevated in FCX and hippocampi of prenatal cocaine-exposed P21 rats. (**A**) Levels of Serine (**S**), Threonine (**T**) and tyrosine (**Y**) phosphorylation on purified native mGluR1 from prenatal saline- and cocaine-exposed P21 rats were determined in immunoprecipitates of immobilized anti-mGluR1 by Western blot using specific antibodies directed against each phospho-epitope. (**B**) pS-mGluR1 levels in immobilized mGluR1 immunoprecipitates of Kreb’s-Ringer (K-R) and 162 nM PMA treated FCX synaptic membrane extracts from prenatal saline- and cocaine-exposed P21 rats. The obtained protein bands were quantified by densitometric scanning of the blots. Data are represented as means ± s.e.m. of the ratios of phosphorylated mGluR1/total mGluR1 optical intensities. *n* = 4 for each group. *p<0.01 comparing the pS-mGluR1 levels induced by PMA vs. K-R in each treatment group. +*p*<0.01 comparing the levels of pS-mGluR1 in prenatal cocaine- to saline-exposed groups by two-tailed Student’s *t* test. #*p*<0.01 comparing the levels of PMA-induced pS-mGluR1 isolated from prenatal cocaine- to saline-treated rats by two-tailed Student’s *t* test. No between-group differences in the levels of mGluR1were detected.

Because mGluR1 is coupled to phospholipase C, we considered PKC as the primary phosphorylating kinase for mGluR1. Incubation of FCX slices from prenatal saline- and cocaine-exposed P21 rats with PKC activator, phorbol 12-myristate 13-acetate (PMA), an approximately 2.5-fold increase in pS-mGluR1 was observed in saline- but not cocaine-exposed tissues (Fig. 5B). To further deduce whether the increased serine-phosphorylated mGluR1 is responsible for the uncoupling of mGluR1 from both G_q/11_ and Homer1, synaptic membranes from prenatal saline- and cocaine-exposed rats were treated with alkaline-phosphatase. Figure 6B illustrates that removal of pS from mGluR1s by alkaline phosphatase treatment in the prenatal cocaine exposed FCX restored Gq/11 and Homer1 coupling to mGluRs to the level observed in saline-treated animals. In addition, incubation of the synaptic membranes from saline-treated rats with recombinant γPKC in the presence 20 µg phosphatidylserine, 1 mM Ca^2+^/162 nM PMA and de-phosphorylated mGluR1 (phosphatase treatment followed by 10 mM NaF and 1 mM Na vanadate), a 2.5–2.7 fold increased in serine phosphorylation of mGluR1 accompanied by a 44.7±2.8% reduction in glutamate-induced coupling to G_q/11_ and a 45.0±3.2–46.2±3.6% decrease in mGluR1- Homer1 association were noted (Fig. 6). These data indicate that reduction in mGluR1 coupling to G_q/11_ and Homer1 in prenatal cocaine-exposed brains is the result of PKC-mediated mGluR1 phosphorylation at the serine sites.

**Figure 6:** Heightened PKC-mediated serine phosphorylation of mGluR1 in prenatal cocaine- exposed brains is responsible for the reduced mGluR1 coupling to G_q/11_ and Homer1. (**A**) Levels of mGluR1 - G_q/11_ and mGluR1 - Homer1 coupling as well as serine-phosphorylated mGluR1 (pS-mGluR1) on purified mGluR1 signaling complexes. FCX synaptosomal membranes from prenatal cocaine- and saline-exposed P21 rats were incubated with either vehicle 100 µM alkaline phosphatase, 30 µM ATP containing Kreb’s-Ringer (K-R) or 162 nM PMA (20 µg phosphoatidylserine). Following completion of dephosphorylation by addition of phosphatase inhibitors, phosphate-free mGluR1 from prenatal saline-treated rats was phosphorylated by recombinant γPKC in the presence of ATP. The reaction was terminated by specific PKC inhibitor, celestrine. The resultant synaptic membranes containing differentially phosphorylated mGluR1 were then incubated with K-R or 1 µM glutamate. The mGluR1 purified by anti-mGluR1 immunoprecipitation was analyzed for phosphoserine by Western blotting. The interaction between mGluR1 and G_q/11_ or Homer1 with different phosphorylation states was assessed by the levels of Gα_q/11_ and Homer1 in the anti-mGluR1 immunoprecipitates by Western blotting. (**B**) Densitometric quantification of mGluR1-associated Gα_q/11_ and Homer1 as well as pS-mGluR1 levels. Data are represented as means ± s.e.m. of the ratios of Gα_q/11_, Homer1 or pS-mGluR1/total mGluR1 optical intensities. *n* = 4 for each group. *p<0.01 comparing the glutamate-induced to basal mGluR1-G_q/11_ complex levels by two-tailed Student’s *t* test. #*p*<0.01 comparing the respected levels in prenatal cocaine- to saline-treated rats. No between-group differences in the levels of mGluR1were detected.

## Discussion

Prenatal cocaine exposure has negative impact on cognitive processing in both humans and animal models as illustrated by reduced attention processing and impairments in motor and language skills as well as associative and discrimination learning, all of which involve excitatory synaptic transmission [26]–[30]. These data suggest that excitatory synapses including those regulated by the mGluR1 are perturbed by cocaine exposure during early brain development. This deficit presumably leads to an altered synaptic plasticity resulting in enduring changes in brain function and abnormal behavior. In support of this possibility, our present data indicate that *in utero* cocaine exposure disrupts mGluR1 coupling to synaptic anchoring protein, Homer1 and signal transducer, Gq/11 protein. By associating with Homer1, mGluR1s cluster in the synaptic membrane. Hence, our data showing that prenatal cocaine exposure uncouple mGluR1 from Homer1 without a detectable change in mGluR1 expression suggest relocation of mGluR1s away from the active glutamatergic synapses to parasynaptic regions. Previously, mGluR and Homer interaction was found to be essential for mGluR signaling mediated long term depression (LTD) [31]. In light of our finding that Homer1 did not directly couple to Gq/11 (data not shown), the reduced mGluR1 - Gq/11 coupling is responsible for the impairment of the mGluR1-mediated phosphoinositide signaling in the prenatal cocaine-exposed brain. The fact that the mGluR1 specific antagonist 3-MATIDA reduced the DHPG-induced IP_3_ accumulation by 65–70% coupled with a 63.4–69% reduction in mGluR1-Gq/11 association suggests that prenatal cocaine may also attenuate mGluR5 signaling.

Concurrent with a reduced mGluR1 signaling shown here, attenuated AMPAR and NMDAR function were also noted in brain tissues from *in utero* cocaine-exposed rodents [5]–[7]. The impaired AMPARs in the prenatal cocaine exposed rat brains was found to be associated with disrupted GluR2/3 - GRIP interaction [6]. These findings indicate that prenatal cocaine profoundly affects the signaling processes mediated by multiple glutamatergic receptors. The fact that activation of mGluR1 rescued the delayed synaptic maturation with impaired AMPAR and NMDAR function in the prenatal cocaine-exposed brains suggests that mGluR1 is a key regulator of the glutamatergic synaptic maturation during brain development [7]. Since mGluR1 is expressed abundantly in cognition- and reward-relevant brain areas including NAc and VTA, a profound reduction in the mGluR1 coupling to Homer1 and Gq/11 in the prenatal cocaine-exposed brain coupled with attenuated signaling is likely to hamper also AMPAR and NMDAR signaling [7], leading to the deficits in cognition and the impaired reward processing seen in animals exposed to cocaine during gestation. This impairment in reward processing is evidenced by studies showing that rabbits exposed to cocaine *in utero* are tolerant to cocaine-induced motor sensitization, which is considered a behavioral correlate of addictive process [32], [33].

The reduced coupling of mGluR1 to Homer1 and Gq/11 is the result of a sustained PKC-mediated phosphorylation of mGluR1 in prenatal cocaine-exposed brains. This observation is reminiscent of our previous report that an increased phosphorylation of D_1A_ dopamine receptors in prenatal cocaine-exposed rabbits results in uncoupling of D_1A_ dopamine receptors from their signal transducer, G_s_ and G_olf_ proteins [26]. A sustained PKC activation indicated by an overwhelming cytosol-to-membrane translocation together with markedly increased association of GRIP with activated PKC-α, -γ and -ζ as well as PKMζ has been reported in prenatal cocaine-exposed brains [6]. This results in a sustained PKC- and Src-mediated phosphorylation of GRIP, the synaptic anchoring protein for GluR2- and GluR3-containing AMPARs thus preventing GRIP from interacting with GluR2/3 [6]. Unlike our previous finding, PKC but not Src mediates mGluR1 phosphorylation since serine phosphorylation is exclusively elevated in mGluR1 of the prenatal cocaine brains. In agreement with our theory that PKC hyperactivation plays a pivotal role in cognitive processing in prenatal cocaine-exposed individuals, excessive PKC activation was found to dramatically impair prefrontal cortex-mediated cognitive functions and increase distractibility [34]. Future experiments are needed to determine whether the reduced mGluR1 - Homer1 - Gq/11 coupling observed in brains of P21 prenatal cocaine-exposed rats is persistent or simply a transient shift in synaptic plasticity during early development. Nevertheless, previous studies conducted by us and others in rabbit indicate that such synaptic plasticity changes are persistent well into adulthood [35]–[37].

In addition to the profound downregulation of the glutamatergic mGluR1, AMPAR and NMDAR function [5], [6] prenatal cocaine exposure has been shown to affect other neurotransmitter systems including dopamine D_1_ receptor - G_s/olf_ coupling [19], [20], [26], GABAergic neurons [38] and the noradrenergic system [39]. Notwithstanding these changes reported to occur in prenatal cocaine-exposed brains, we propose that hyper-activation of PKC resulting in sustained phosphorylation of mGluR1s and the consequent uncoupling of mGluR1 from Homer1 and Gq/11 elucidated here may be one of the prominent events underlying prenatal cocaine-induced cognitive impairment. Moreover, both our previous and current data suggest that blocking excessive PKC translocation, a primary PKC activation mechanism, may be effective in preventing/reversing prenatal cocaine from promoting protracted deficits in AMPAR- and mGluR- regulated neurotransmission [6], [40]. In this regard, therapeutic agents such as lithium and valproate that block PKC translocation without directly interfering with its enzymatic activity [41] may have therapeutic value in maintaining adequate mGluR1-regulated synaptic activity in subjects exposed to cocaine during gestation.
